The article "Evaluation of Uterotonic Activity, Acute Oral Toxicity, and Phytochemical Composition of Uvariodendron anisatum Verdc. Root Extracts" was published in 2022. Journal: Evid Based Complement Alternat Med.

# Evaluation of Uterotonic Activity, Acute Oral Toxicity, and Phytochemical Composition of *Uvariodendron anisatum* Verdc. Root Extracts

**DOI:** 10.1155/2022/7393537

**Published:** 2022-08-25

**Authors:** Kanji Benson Muthee, Timothy E. Maitho, Laetitia Wakonyu Kanja, Jared Misonge Onyancha

**Affiliations:** ^1^Department of Public Health, Pharmacology & Toxicology, Faculty of Veterinary Medicine, University of Nairobi, P.O. Box 29053-00625, Nairobi, Kenya; ^2^Department of Pharmacognosy, School of Pharmacy, Mount Kenya University, P.O Box 342-0100, Thika, Kenya

## Abstract

Over 80% of cultural societies in low-income countries use plant preparations in traditional medicine with unknown potency and safety profiles. *Uvariodendron anisatum* root extracts are used by some Kenyan herbalists. However, the claims of the plant to remove retained placenta during birth have remained uninvestigated. Therefore, the current study evaluated its uterotonic activities. Acute toxicity in Wistar rats and the phytochemical composition of the plant were also studied. The plant was collected from Embu County in Kenya. The water and ethanol extracts were prepared by maceration. Uterine strips were isolated from primed mature female Wistar rats and used to study the uterotonic activities of the extracts. De Jalon's solution and oxytocin were used as negative and positive controls, respectively. Acute oral toxicity studies were done following the OECD 423 guideline and phytochemical screening were based on standard phytochemical procedures. The study met all the approval requirements before commencement. Data obtained from the uterotonic activity were analysed by using GraphPad Prism Version 8.0.1 software and expressed as a percentage increase or decrease of mean as mean ± SEM relative to the controls. The findings of acute oral toxicity were expressed using LD_50_. Additionally, the phytochemical components of the *U. anisatum* were tabulated. The uterotonic effect of *Uvariodendron anisatum* root water extract was higher than that of ethanol extract. A single dose of the *Uvariodendron anisatum* root water extract at 2000 mg/kg did not cause mortality in the tested Wistar rats. Besides, there were no changes in hematological and biochemical parameters. The extracts did not reveal changes in the gross morphology of the liver, kidney, heart, and lung of the tested Wistar rats. However, the histopathological studies of *Uvariodendron anisatum* root water extracts exhibited toxicity in the liver, kidney, and lung tissues of Wistar rats at a concentration of 2000 mg/kg. Alkaloids, glycosides, saponins, phytosterols, terpenes, proteins, phenols, and oils were recorded in *Uvariodendron anisatum.* The findings from this study provided scientific evidence which is useful in validating the use of *Uvariodendron anisatum* extracts in the stimulation of the uterus during birth.

## 1. Introduction

Medicinal plants continue to be used in traditional complementary alternative medicine for the health care of pregnant women in many low- and middle-income countries globally [1]. Health has a central place in the Nations Sustainable Development Goal (UN SDG 3) to “ensure healthy lives and promote wellbeing for all at all ages,” where maternal and child health is underpinned by targets 3.1 and 3.2 and cover a wide spectrum of World Health Organization's work [2]. In 2015, the inclusion of Universal Health Coverage (UHC) in the SDGs as target 8 under SDG 3.8 provide an opportunity to ensure that all people and communities have access to the healthcare services that they want and need without suffering financial hardship [3]. Primary health care is key to the attainment of UHC which is fundamental to attaining SDG 3.

Plants used in complementary medicines have remained significant in primary health care throughout humanity's history [4]. Various cultural societies have plant-based medicines which manage delivery-associated complications in alternative medicine systems [5–7]. Some of the medicinal plant preparations known to have uterotonic activities are reported to decrease post-partum haemorrhage (PPH) and other birth-related illnesses in Africa. Post-partum haemorrhage is the principal reason for maternal mortalities, as well as morbidities in developing states. Therefore, medicinal plant preparations with proven efficacy and safety may prove beneficial in reducing maternal deaths. The current study seeks to evaluate the uterotonic activity of *Uvariodendron anisatum* root extracts. Acute oral toxicity in Wistar rats and the phytochemical composition of the plant were also studied. *Uvariodendron anisatum* (*Annonaceae*) has been recorded to have gynecological benefits in some Kenyan communities' traditional medicine systems [8–10]. The current findings from the research provide a platform for validation of the use of the plant in traditional medicine.

## 2. Materials and Methods

### 2.1. Plant Collection, Identification, and Preservation

The roots of *Uvariodendron anisatum* (Annonaceae) were collected with the assistance a of local herbal practitioner from Kianjiru Hills in Mbeere South Subcounty in Kenya. A voucher specimen was prepared and later identified and authenticated by a taxonomist at the National Museums of Kenya, Botany Department. The identity of the plant specimens was further confirmed at the Department of Land Resource, Management, and Technology (LARMAT), at the University of Nairobi. The sample was assigned voucher number BMK02/17/03/2021, it was deposited at the East Africa Herbarium and a duplicate was stored at the University of Nairobi Herbarium.

### 2.2. Preparation of Extracts

#### 2.2.1. Ethanol Extracts

The collected roots of *Uvariodendron anisatum* were cut into small pieces and were spread on the bench to dry at room temperature and pressure. The dried roots were ground into coarse powder using a hammer mill and were extracted by maceration using ethanol. Briefly, two hundred grams of the powdered plant materials were soaked in 250 millilitres of 80% ethanol in a 1000 mL flat-bottomed flask for 48 hours [11]. The root ethanol extract was filtered using Whatman paper No.1 and thereafter reduced by a rotary evaporator at 35°C followed by complete drying using an oven at 40°C [12].

#### 2.2.2. Water Extracts

Water extract of *Uvariodendron anisatum* roots was prepared by freeze-drying. Briefly, one hundred grams of *Uvariodendron anisatum* root powder was boiled in 1 litre of distilled water by using a boiling flask for 1 minute. The resulting decoction was left to cool and then filtered using Whatman paper No.1. The primary filtrate was centrifuged at 3000 rpm for 10 minutes and the supernatant was filtered for a second time using sintered glass. The extract was then lyophilized and the water extracts which were obtained were weighed, labelled, and kept at 4°C [13].

#### 2.2.3. Working Extract Solutions

Ethanol and water extracts were reconstituted in De Jalon's physiological salt solution [13]. De Jalon's physiological salt solution was used to provide the needed organ bath conditions at a capacity of 40 ml in concentrations of 4.0 mg/ml, 2.0 mg/ml, 1.0 mg/ml, and 0.5 mg/ml.

### 2.3. Assay for Uterotonic Potency

#### 2.3.1. Experimental Animals

Mature female Wistar rats which were four months old and weighed 200 ± 5 g were used in this study. A total of 7 rats were obtained from the University of Nairobi, Department of Public Health Pharmacology and Toxicology following random selection. The rats were kept in cages in an air-conditioned room at 22 ± 2°C and 60% relative humidity [14].

Untreated wood shavings were used as beddings and were changed daily. The experimental animals were exposed to 12 hours of light and 12 hours of the dark cycle. The rats were fed with commercial rat pellets which were purchased from Unga Feeds Limited in Nairobi, Kenya. The Wistar rats had free access to clean water *ad libitum* [15]. All the rats were humanely handled as provided for by the Faculty of Veterinary Medicine Biosafety, Animal Use, and Ethics Committee guidelines and allowed to acclimatize for one week before the study started.

#### 2.3.2. Preparation of Uterine Tissues

Wistar rats were pre-treated by using diethylstilbesterol in *Arachis* oil (1 mg/kg, i.p.) for 24 hours preceding the actual experiment to induce the oestrus phase cyclicity [16]. The rats were then sacrificed humanely using phenobarbital as described by Goodies et al. [17]. Thereafter, dissection of the rats was done to open the abdominal cavity and the two horns of the uterus were carefully removed and they were placed in a petri dish containing warm and aerated De Jalon's solution. All connective tissues on the uterine horns were removed in the preparation of the horns which were used for uterotonic activity assay.

#### 2.3.3. Uterotonic Activity of Extracts

Uterine strips 2 cm long were cut from the uterine horns and each strip was attached vertically within the organ bath comprising 40 ml De Jalon's solution composed of 0.5 g glucose, 9.0 g NaCl, 0.42 g KCl, 0.24 g CaCl_2_, 4.5 g sucrose, 0.142 g NaH_2_PO_4_, as well as 2.1 g NaHCO_3_ reconstructed in a litre of purified water. The mixture was then aerated using a blend of 5% CO_2_ and 95% O_2_ [18]. The organ bath temperature was maintained at 37 ± 0.5°C to ensure tissue viability [13]. The upper end of the uterine segment was hooked to an isometric force transducer (ML500/A, AD device) which was supplemented by using Power Lab data acquisition equipment (Power Lab 8/30) [14]. The frequency of uterine contractions (number of peaks recorded) and amplitude of contraction (in microvolts) were recorded and analysed using Chart 5 software supported by windows. The experiments were done in triplicates, and each experiment was supplemented using a negative control (De Jalon's solution). The study also included a positive control (oxytocin IU) in order to allow comparison [13, 14].

#### 2.3.4. Contractions for Negative and Positive Controls

The mounted uterine strips were allowed 30 minutes to recover and stabilize in De Jalon's solution. The contractions of the isolated uterine strips were recorded for 10 minutes. These initial contractions were taken as the negative control recordings. After 10 minutes of negative control contractions, 1.0 ml of oxytocin (10 IU) was introduced and the isometric contractions were recorded for 10 minutes which were considered as a positive control.

#### 2.3.5. Contraction Activity of Extracts On an Isolated Wistar Rat Uterus Strip

Fresh uterine horns were prepared as described previously. After the first 10 minutes of negative control contractions, 1 ml of 0.5 mg/ml of the *U. anisatum* was introduced to the organ bath. Isometric contractions were recorded for 10 min followed by washing the strip three times with De Jalon's solution. A 30-minute uterine recovery time was allowed to normalize the contractions. Subsequently, the procedure was repeated with the 1.0 mg/ml, 2.0, and 4.0 mg/ml. The experiments were done in triplicates by employing unused strips in every dosage scale as well as rinsing the tissues well before each assay of the different extract dose [13]. The frequency and amplitude of uterine contractions was calculated and recorded.

### 2.4. Acute Oral Toxicity

Mature female Wistar rats, aged four months and weighing 200 ± 5 g, were used to evaluate acute oral toxicity of *U. anisatum* roots extracts. The process involved randomly selecting rats and grouping (*n* = 3) using picric acid markings. The selected rats were kept separately for five days in polycarbonate cages to allow laboratory acclimatization before conducting the test.

#### 2.4.1. Lethal Dose

The universal protocol and instructions for severe oral toxicity identified by the Organization for Economic Co-operation and Development (OECD) Guideline 423 [19, 20] was used. Prior to treatment, the process entailed fasting experimental rats overnight and weighing. Additionally, a single dosage of the test extract was administered using gavage at 300 mg/kg and signs of toxicity were observed up to 24 hours. A repeat of 300 mg/kg was administered to another set of three experimental rats. Thereafter, a higher dose of 2000 mg/kg body weight was administered to another group of three experimental rats. A repeat of 2000 mg/kg body weight dose was administered to a separate group of three experimental rats. Normal saline was used for the control group. Health parameters were observed and recorded chronologically for 2 weeks as indicated by the OECD/2001/423. Besides, behavioural responses, general appearance haematological, and biochemical effects of the plant extracts were evaluated by using standard methods [21, 22].

#### 2.4.2. Haematological and Serum Biochemistry Studies

The effects of *Uvariodendron anisatum* root water extracts were done following the method described by Antai et al. [23] with slight modifications. At the end of each experiment (at 15^th^ day for acute oral toxicity), 1.5 ml blood was collected from the lateral veins of restrained Wistar rats using a disposable syringe. One millilitre of the collected blood was put in tubes containing ethylenediamine tetraacetic acid (EDTA) and was used for the analysis of haematological parameters of the white blood cell (WBC). The differential white blood cell count by microscopic blood smear. Briefly, one drop of blood was used to make a smear on a microscopic slide which was followed by air drying for one minute to prevent haemolysis. The smeared and dry microscopic slides were then stained by Giemsa for 30 minutes and pH of 7.2. The various types of white blood cells were counted at 100x (100 times) magnification and the percentage of neutrophils, lymphocytes, eosinophils, and basophils of each type was calculated [24].

On the other hand, 0.5 millilitres of the collected blood were placed in nonheparinized tubes and were left for 15–20 minutes at room temperature to promote blood coagulation. The blood sample was then centrifuged at 5000 rpm for 20 minutes at 40°C and the serum which was obtained serum was put in Eppendorf tubes and transported in a cool box containing ice packs to Lancet Laboratories at Nairobi (Kenya) where the contents of urea, creatinine, alkaline phosphatase (ALP), alanine transaminase (ALT), and aspartate aminotransferase (AST) were quantified. Immediately after blood collection, the rats were sacrificed by cervical dislocation and the liver, kidney, lung, and heart were harvested for histopathological studies.

#### 2.4.3. Histopathological Studies

The method was described by Loha et al. [25] with modifications. The liver, kidney, lung, and heart of 2 mm thick sections were taken randomly and were fixed in 10% neutral buffered formalin (NBF) overnight at room temperature. After fixation, the tissue sections were washed with water to remove excess fixatives for six hours and dehydrated with graded alcohol baths of 50%, 70% for two hours, 90% for two hours, 100%, 100% for one and half hours in each case and finally, in 100% alcohol for twelve hours. The dehydrated tissues were cleared in two steps of dealcoholisation using xylene for one and half hours and two and half hours, respectively.

Infiltration of the tissues was done using molten paraffin wax at 62°C for thirty minutes. Finally, the tissues were embedded in paraffin wax in square metal plates (cassettes) forming tissue blocks, whereby each tissue block was labeled and stored at room temperature till the time they were sectioned. The tissue blocks were sectioned in ribbons at a thickness of 5 *μ*m using Leica microtome (Leitz Wetzlar). The ribbons of the sections were collected at every 5^th^ section and put onto the surface of warm water bath of temperature of 40°C. The floating ribbons were mounted onto clean slides. The slides containing paraffin wax were arranged within the slide holder and placed in an oven with temperature of 40°C for about 20 minutes so as to fix the tissue to the slides and allowed to cool at room temperature for 30 minutes.

Thereafter, the mounted sections were stained regressively with the routine Harris Haematoxylin Eosin staining technique. Briefly, two series of coupling jars were prepared, one for paraffin removal and hydration and the other for dehydration and clearing. Sections were placed in xylene I for 5 minutes and xylene II for 2 minutes again to remove the paraffin from tissue and hydrated by treating them with decreasing concentrations of 100%, 100%, and 95% alcohol for two minutes each, 70% of alcohol for three minutes and 50% alcohol for five minutes. The tissue sections were washed with tap water for five minutes and stained regressively with Harris Haematoxylin for 6 minutes and then washed under running tap water for five minutes. The slides were immersed in acidic alcohol for differentiation and controlling over stained Haematoxylin for 1 second and then put in bluing solution (sodium bicarbonate) until they became blue. After bluing, the slides were counter stained with Eosin for 20 seconds and then washed in tap water for two minutes. The sections were dehydrated with increasing alcohol concentration of 50%, 70%, 95%, 100%, and 100% for two minutes each. The dehydrated sections were cleared with xylene I and xylene II for three minutes each and were permanently mounted on microscopic slides using dibutylphthalate polystyrene xylene (DPX) and cover slips and then observed under a light microscope for the investigations of any histological change, thereby the histology of the treated groups was compared with histology of the control group. After examination, photomicrographs of selected samples of the liver, kidney, lung, and heart section from both the treated and control rats were taken under a magnification of ×400 objective using (Olympus CX21).

### 2.5. Phytochemical Screening

The analysis of the phytochemical groups of compounds, namely, plant sterols, terpenoids, diterpenes, phenols, flavonoids, glycosides, fats, and volatile oils of water and ethanol extracts of *Uvariodendron anisatum* root were done using standard phytochemical screening procedures described by Houghton and Raman, [26]; Harborne, [27] as modified by Moriasi et al. [28]. The tests were performed in triplicates in order to ensure the results' accuracy and were examined by visual observations.

#### 2.5.1. Test for Alkaloids

Two tests, namely, Mayer's and Dragendorff's tests, were done in order to detect alkaloids in the extracts. Approximately, 0.1 g of water and ethanol extracts of *Uvariodendron anisatum* root were mixed with 5 ml of 1% HCl in separate test tubes, respectively; each mixture was warmed and then filtered through Whatman filter paper No.1. Two drops of Mayer's reagent (mercuric potassium iodide) were added to 2 ml of water and methanol extracts. The appearance of a cream-coloured precipitate indicates the presence of alkaloids. Dragendorff's test was carried out by adding two drops of Dragendorff's reagent (potassium bismuth iodide solution) to 2 ml of the filtered water and ethanol extracts in separate test tubes. A reddish-brown precipitate indicates the presence of alkaloids [11].

#### 2.5.2. Test for Phenolics

Approximately, 100 mg of the aqueous and ethanol extracts of *Uvariodendron anisatum* root were measured and put into separate test tubes and 10 ml of 70% ethanol were added. The mixtures were boiled by using water for five minutes. The extracts were then cooled, and they were filtered through Whatman filter paper No.1. Five drops of 5% of ferric chloride were added into 2 ml of each respective extracts. The formation of a green precipitate indicates the presence of phenols [12].

#### 2.5.3. Glycosides

*(1) Modified Borntrager's test*. Approximately, 200 mg of the aqueous and ethanolic extracts of *Uvariodendron anisatum* root were dissolved in 5 ml of 5% H_2_SO_4_. Three millilitres of the mixtures were filtered into separate test tubes and thereafter 2 ml of ferric chloride were added to the test tubes and shaken. The solutions were heated on a water bath for 10 min. The extracts were filtered while hot using Whatman filter paper No.1. The filtrates were allowed to cool and then equal volume of dichloromethane was added and gentle shaken. The organic layer was separated and washed with 5 ml of dilute ammonia solution. A rose-pink to cherry-red colour in the ammoniacal layer indicated the presence of anthraquinone [12, 29].

*(2) Keller–Killiani test*. Glacial acetic acid (4.0 ml) solution with 1 drop of 2.0% FeCl_3_ mixture was added to the 10 ml aqueous and ethanol extracts of *Uvariodendron anisatum* root in separate test tubes. One millilitre of concentrated sulphuric acid was added to the mixture and a reddish brown ring formed between the layers which progressively turned blue indicated the presence of steroidal glycosides with deoxy sugars [12].

*(3) Kedde test*. One millilitre of 2% solution of 3,5-dinitrobenzoic acid in 95% alcohol was added to the 2 ml of the aqueous and ethanol extracts of *Uvariodendron anisatum* root. The solution was made alkaline with 5% sodium hydroxide. The appearance of a purple-blue colour indicates the presence of unsaturated lactone ring in cardenolides [12, 30].

#### 2.5.4. Test for Flavonoids (Sodium Hydroxide Reagent Test)

Approximately, 0.1 g of the aqueous and ethanolic extracts were warmed in 10 ml of 70% ethanol and thereafter hydrolysed by 10% hydrochloric acid. Sodium hydroxide (10%; 1 ml) was added to the mixture and the appearance of yellow colour was a positive test for the presence of flavonoids [31, 32].

#### 2.5.5. Test for Triterpenoids (Salkowski's Test)

Approximately, 2 mg of the aqueous and ethanol extracts of *Uvariodendron anisatum* root were dissolved in 1 ml of chloroform and then shaken gently. Five drops of concentrated sulfuric acid were added along the side of the test tube. A reddish-brown colour which was formed at the interface indicated terpenoids [29, 33].

#### 2.5.6. Phytosterols (Lieberman Test)

In this study, 0.1 g of water and ethanol extracts from *Uvariodendron anisatum* root were dissolved in 2 ml acetic anhydride and were heated to the boiling point. The mixtures were filtered by using Whatman filter paper No.1 to separate test tubes. One drop of concentrated sulphuric acid was added slowly along the sides of the test tube. An array of colour change ranging from red to blue showed the presence of phytosterols [33, 34].

#### 2.5.7. Test for Saponins (Froth Test)

About 0.1 g of the aqueous and ethanol extracts of *Uvariodendron anisatum* root were added to 10 ml of distilled water in separate test tubes, respectively. The mixtures were boiled for 10 minutes and they were filtered using Whatman filter paper No.1. A mixture of 3 ml distilled water and 5 ml of the filtrate were agitated vigorously for 15 seconds and left to stand for 10 minutes. The formation of a 1 cm layer of a stable honeycomb like froth which persisted for about 3 minutes was an indication of saponins [12].

#### 2.5.8. Detection of Diterpenes (Copper Acetate Test)

Two grams of *Uvariodendron anisatum* powder were extracted using five millilitres of water in a test tube. The extract was filtered using a Whatman No.1 filter paper. Three drops of copper acetate solution were added into one millilitre of the extract in a test tube. The formation of an emerald green colour was indicative of the presence of diterpenes [35].

#### 2.5.9. Test for Proteins (Xanthoproteic Test)

One ml of the extracts was treated separately with two drops of conc. HNO_3_; the formation of a yellow precipitate indicates the presence of proteins [36, 37].

#### 2.5.10. Test for Fixed Oils (Spot Test)

Two milligrams of *Uvariodendron anisatum* root dry powder and extracts were pressed between two filter papers. Oil stain on the paper indicates the presence of fixed oils [38].

#### 2.5.11. Test for Volatile Oils

Fifty grams of a powdered material (crude drug) is taken and subjected to hydrodistillation. The distillate is collected in graduate tube of the assembly, wherein the aqueous portion automatically separated out from the volatile oil [39].

### 2.6. Data Analysis

The mean frequency (rate) and mean amplitude (force) of uterine contractions were analysed from the chart recordings. Mean frequency was the number of contractions over a period of ten minutes divided by the 10 minutes and this was the number of peaks recorded. The mean amplitude or force was the mean height in microvolts (*μ*V) of the peaks produced over the 10 minutes. By comparing the mean frequency and mean amplitude of contraction for the control and test groups, it was possible to determine whether the extract increased, reduced, or did not cause any effect in terms of mean frequency and mean amplitude of uterine contraction. Uterotonic activity was expressed as a percentage increase or decrease in mean ± standard error of the mean (SEM) relative to the controls, using the formula described by Wairimu et al. [14].

(1) $$\begin{array}{c} \text{Percentage contractions}=\left(\frac{F/At-Fc}{Fc}\right)\times 100, \end{array}$$

where *F*/*At* = frequency or amplitude after treatment and *Fc* = control contractions.

GraphPad Prism Version 8.0.1 software was used for analysis of data. Descriptive analysis of the mean frequency and mean amplitude of uterine contractions was done by using one-way ANOVA. At the same time, levels of significance were established using *P* values at *P* < 0.05 (^*∗*^); *P* < 0.01 (^*∗∗*^); and *P* < 0.001 (^*∗∗∗*^). Moreover, a post hoc Tukey's multiple comparison evaluation was conducted in order to analyse statistical differences among groups.

The results from acute oral toxicity which included parameters of wellness were tabulated. The dose that killed 50% of the experimental rats (LD_50_) were recorded and interpreted according to OECD Guideline 423 [20]. Data for qualitative analysis of phytochemicals were also summarized using tables.

### 2.7. Ethical Consideration

The authority to conduct the study was requested from the Faculty Biosafety, Animal Use and Ethics Committee (BAUEC). The permission to conduct the study was granted by BAUEC in a letter with reference number of FVMBAUEC/2021/295. Research authorization was also obtained from National Commission for Science, Technology, and Innovation (NACOSTI) with a license number NACOSTI/P/21/11761. The obtained data were stored in a laptop and confidentiality was maintained throughout the study.

## 3. Results

### 3.1. Isolated Wistar Rat Uterine Strip Contractility

The uterine muscular contraction against resistance in which the length of the muscle was 2 cm (isometric contractions) was observed to increase with increased concentrations of crude extracts or standard drug (oxytocin 10 IU) under the current study. The contractions were dose-dependent and contractility of the uterine strip increased up to a maximum concentration of 1 mg/ml, except for the *Uvariodendron anisatum* ethanol extract that revealed maximum contractility at 2 mg/ml.

### 3.2. Effects of *U. anisatum* Root Extracts on the Mean Force and Mean Frequency of Wistar Rats Uterine Strip Contractions

The water and ethanol extracts from *Uvariodendron anisatum* root revealed a dose-dependent effect on percentage mean force of the uterine contractions (Table 1). There was a notable increase of percentage mean force on the contractions of the uterine strip by 27.633 ± 0.711 at 0.5 mg/ml which reached a maximum effect by 95.228 ± 2.013 at 1 mg/ml of the water extract. A decline of percentage mean force effect was detected from 95.228 ± 2.013 to 84.897 ± 1.631 and 66.320 ± 1.631 at 2 mg/ml and 4 mg/ml, respectively, for the water extract. There was an increase of percentage mean force of 67.477 ± 0.826, 69.304 ± 0.832 and to a maximum of 82.145 ± 0.055 at concentrations of 0.5 mg/ml, 1 mg/ml, and 2 mg/ml, respectively, for the ethanol extract. Thereafter, the percentage mean force decreased to 44.749 ± 1.065 at a concentration of 4 mg/ml. A comparison of effects of *Uvariodendron anisatum* root water and ethanol extracts concentrations on the mean force of Wistar rats uterine strip contractions revealed significant difference with *P* < 0.001^*∗∗∗*^ at 0.5 mg/ml, 1 mg/ml, and 4 mg/ml whereas there was no significant difference at concentration 2 mg/ml (Figure 1).

The percentage mean frequency of uterine contractions of water extract of *Uvariodendron anisatum* root was 39.996 ± 2.508 at a concentration of 0.5 mg/ml. At a concentration of 1 mg/ml, the percentage mean frequency increased to maximum percent of 78.140 ± 2.432. A decline of the percentage mean frequency from 78.140 ± 2.432 to 34.339 ± 3.485 and 22.583 ± 1.764 was observed at concentrations of 2 mg/ml and 4 mg/ml, respectively. The ethanol extract, also revealed increasing percentage mean frequency of uterine contraction from 18.099 ± 2.970 to 85.429 ± 2.970 from 0.5 mg/ml to 2 mg/ml and later a decline in percentage frequency to 69.461 ± 1.485 at 4 mg/ml (Table 1). A comparison between percentage mean frequency of ethanol and water extract of *Uvariodendron anisatum* root at different concentrations revealed significant difference *P* < 0.001^*∗∗∗*^ at 0.5 mg/ml, 1 mg/ml, 2 mg/ml, and 4 mg/ml (Figure 2). The ethanol extracts revealed significantly high percentage mean frequency at concentrations 0.5 mg/ml, 1 mg/ml, and 2 mg/ml. The effect of *Uvariodendron anisatum* root water extract on the frequency of uterine contractions was higher than that of ethanol up to concentration of 2 mg/ml after which it dropped (Figure 2).

### 3.3. Toxicity of *U*. *anisatum* Root Extracts on Female Wistar Rats

The evaluation of toxic effects of a single dose of water and ethanol extracts of *Uvariodendron anisatum* root extracts administered orally to Wistar female rats was assayed. The lethal dose (LD_50_), behavioural changes, and changes in blood parameters revealed that all the doses used in the current study, from 300 and 2000 mg/kg body, were nontoxic to the female Wistar rats.

#### 3.3.1. Acute Oral Toxicity of *Uvariodendron anisatum* Root Extracts on Mortality of Female Wistar Rats

In the current study, all the Wistar female rats in the treatment group survived after administration of single dose at 300 and 2000 mg/kg of the water and ethanol extracts from *Uvariodendron anisatum* root extracts. Therefore, there were no mortalities that were observed even after administration of the highest possible acceptable single dose of 2000 mg/kg body orally to all groups. In addition, the behavioural responses and general appearance of the female Wistar rats which were treated with single dose of *Uvariodendron anisatum* root extracts are recorded in Table 2. None of the female Wistar rats treated with single doses of *Uvariodendron anisatum* root extracts showed remarkable changes in clinical observations during the study period.

#### 3.3.2. Toxic Effects of the *Uvariodendron anisatum* Root Water Extract on Blood Biochemical Parameters

Table 3 indicates the mean ± SEM of the observed values which were obtained from liver function assessments, namely, alkaline phosphatase (ALP), alanine aminotransferease (ALT), aspartate aminotransferase (AST) and kidney function assessments which were Blood urea and creatinine blood tests. The mean values of the estimated blood parameters from duplicate readings were within the normal ranges of both control group and extracts treated groups (Table 3).

#### 3.3.3. Toxic Effects of *Uvariodendron anisatum* Root Water Extract on Some Hematological Parameters

In this study, the data of the observed toxic effects of *Uvariodendron anisatum* root water extracts on blood plasma are recorded in Table 4. The differential count of white blood cells from both the control and extracts treated rats (2000 mg/kg body weight), indicated that neutrophils, lymphocytes, eosinophils, and basophiles were within the normal range. *Uvariodendron anisatum* root water extracts revealed percentage composition of white blood cells at normal ranges too. The percentages for neutrophils were 17.0 ± 3.6%, lymphocytes 81.0 ± 4.7%, eosinophils 2.0 ± 1.15%, and basophiles 0%.

#### 3.3.4. Toxic Effects of the *Uvariodendron anisatum* Root Water Extract on Wistar Rat Organs

The gross morphology of the organs in the current study, liver, kidney, heart, and lung did not exhibit pathological lesions. However, light microscopic examination of sections of the studied organs which were stained with Haematoxylin and Eosin at magnification of 400x (400 times) revealed some abnormalities as shown in Figures 3–5 for the Wistar rats in the test groups.

The *Uvariodendron anisatum* root water extract exhibited histopathological changes in the liver tissues of the Wistar rats which were treated with 2000 mg/kg body weight (Figure 3). Letter (*C*) in a photomicrograph (b) indicates that *Uvariodendron anisatum* root water extracts caused congestion of hepatic blood vessels. This observation was considered abnormal compared to the one for the photomicrograph (a) which represents the tissue from the control group of Wistar rats.

Figure 4 shows histopathological changes caused by *Uvariodendron anisatum* root water extracts in the kidney sections of the Wistar rats. Photomicrographs from the control group (a) while IV represent abnormalities in the kidney tissues after oral administration of a single dose of the *Uvariodendron anisatum* root water extract at 2000 mg/kg body weight to the test group. The letter (*T*) and the star in photomicrograph (b) revealed the observed diffuse hemorrhages in the interstitial spaces and focal hemorrhages in the kidney sections respectively. The results for the control group in the current study revealed diffuse congestion of blood vessels (*C*) and infiltration of interstitial spaces with polymorphonuclear cells (arrow) and in this case were considered histological artifacts.

Figure 5 shows the histopathological effects of *Uvariodendron anisatum* root water extracts in the heart sections. The photomicrographs in (a) for control group and (b) for the group which was treated with 2000 mg/kg body weight of the *Uvariodendron anisatum* root water extract. The observation made on the test groups did not show histopathological differences when compared to the control group. Therefore, the water extract of the *Uvariodendron anisatum* root did not have any observable effects in the heart sections.

Figure 6 shows the histopathological effects of the *Uvariodendron anisatum* root water extract in the lung sections. The photomicrographs in (a) for the control group and (b) for groups which were treated with 2000 mg/kg body weight of the *Uvariodendron anisatum* root water extract. The observed congestion of blood vessels represented by letter (*C*) and polymorphonuclear cells infiltration (arrow) of bronchioles in photomicrograph (b) revealed lung injury caused by the *Uvariodendron anisatum* root water extract at 2000 mg/kg body weight.

### 3.4. Phytochemical Composition of *U*. *anisatum* Extracts

The results of phytochemical screening of *Uvariodendron anisatum* powders and extracts are shown in Table 5. The *U. anisatum* root powder and extracts revealed the presence of alkaloids, saponins phytosterols, glycosides, terpenoids, diterpenoids, fats, volatile oils, proteins, and phenolics.

## 4. Discussion

The most important finding of the current study was the scientific evidence to support the efficacy of *Uvariodendron anisatum* root extracts in inducing uterine contractions. It was found that both the ethanol and water extracts of the *Uvariodendron anisatum* root had uterotonic activities. It was found that the water and ethanol extracts of the *Uvariodendron anisatum* root demonstrated uterotonic activity on the uterine strips of Wistar rats. The results of the uterotonic effects of water extract of *Uvariodendron anisatum* are consistent with the findings reported by Misonge et al. [40]. Studies of the other plants in the *Annonaceae* family are reported as useful crude drugs with uterotonic drugs [41]. The root extracts of *Uvariodendron kirkii* (*Annonaceae*) has also revealed uterotonic activities on the uterine strips [14].

The water and ethanol extracts of *Uvariodendron anisatum* root were classified in the range of category five (LD_50_ > 2000 mg/kg body weight) according to the globally harmonised classification system for chemical substances and mixtures [20]. The absence of animal mortalities in the extract treated groups at highest dose of 2000 mg/kg body weight was interpreted as LD_50_, which is a toxic dose which kills half of the experimental animals was more than 2000 mg/kg body weight. This indicates that single oral dose of the water and ethanol extracts of the *Uvariodendron anisatum* root were nontoxic to Wistar rats. The acute oral toxicity findings of the ethanol and water extracts of the *Uvariodendron anisatum* root on Wistar rats were reported for the first time in this study. Literature reports indicate that the methanol and water extracts of *Uvariodendron anisatum* root are also nontoxic to Wistar rats following administration of a single oral dose at 2000 mg/kg body weight [42]. In addition, there were no observable clinical signs of toxicity after single dose of administration of 2000 mg/kg body weight of the water and ethanol extracts of the *Uvariodendron anisatum* root.

The report of the current study indicates that the water extracts of the *Uvariodendron anisatum* root extract did not show any variations from the normal range values. The study indicated that the extracts did not alter the liver or the kidney functions. Additionally, there were no toxic effects of water extracts of the *Uvariodendron anisatum* root on the studied white blood cell composition.

The phytochemical compounds which were detected in the present study are associated with the biological activities which are used to manage various conditions in human beings. Other early reports are consistent with the current study where the presence of glycosides, alkaloids, phytosterol, phenols, flavonoids, saponins, and triterpenes in some extract of are reported [40]. Some of the phytochemicals which were reported in the current study as phenolics, diterpenes, glycosides, steroidal saponins, plant sterols, and proteins have been described to be responsible for the uterotonic activity of the plants in which they are contained [1].

## 5. Conclusion

It was concluded that *Uvariodendron anisatum* root extracts have uterotonic activity on the isolated uterine strips of Wistar rats. This was demonstrated by the increase in percentage mean force and mean frequency following the increase of the administered dose and compared with the standard (Oxytocin 10 IU). The extracts of the *Uvariodendron anisatum* root were nontoxic when given orally as a single dose because there were no fatalities at doses of 2000 mg/kg body weight. The uterotonic activity of *Uvariodendron anisatum* root extracts can be explained by the presence of phytochemicals which were detected in this study. The study has provided a scientific understanding of the safety and efficacy of *Uvariodendron anisatum* extracts. The findings provided preliminary information to validate uterotonic and safety profile of *Uvariodendron anisatum*. Therefore, this information can act as a guide for the rational use of *Uvariodendron anisatum* extracts by traditional midwives in the course of assisting mothers with retained placenta during birth.

## 6. Recommendation

The findings of the present study show that the use of *Uvariodendron anisatum* water preparations by traditional medicine practitioners for a long time without scientific data are validated partially using these results. Additionally, bioactivity guided isolation and identification of phytochemicals which are responsible for the uterotonic activity should be studied. Subchronic and chronic toxicity studies to establish the toxic effects of *Uvariodendron anisatum* root extracts following multiple doses and a long time of exposure should be conducted. The study on mode of actions of the extracts of the *Uvariodendron anisatum* root should also be conducted.

## Figures and Tables

**Figure 1:** Effects of water and ethanol extracts of the *U. anisatum* root on the mean force of uterine contractions.

**Figure 2:** Effects of *U. anisatum* root water and ethanol extract concentrations on percentage mean frequency of uterine contractions.

**Figure 3:** Photomicrograph of the liver section from Wistar rats in the acute oral toxicity study from control group (a) and rats which were treated with 2000 mg/kg (groups (b)) of *U. anisatum* root water extracts.

**Figure 4:** Photomicrograph of the kidney section from Wistar rat in acute oral toxicity study: from control group (a) and rats which were treated with 2000 mg/kg (groups (b)) of *U. anisatum* root water extracts.

**Figure 5:** Photomicrograph of the heart section from Wistar rats in the acute oral toxicity study from control group (a) and rats which were treated with 2000 mg/kg (groups (b)) of the *U. anisatum* root water extract.

**Figure 6:** Photomicrograph of the lung section from Wistar rat in the acute oral toxicity study from control group (a) and rats which were treated with 2000 mg/kg (groups (b)) of *U. anisatum* root water extract.

**Table 1:** Effects of *U. anisatum* root extracts concentrations on the mean force and frequency of uterine contractions.

Extract or drug concentration	*% Mean force* *±* *SEM*		*% Mean frequency* *±* *SEM*	
	Water	Ethanol	Water	Ethanol
0.5 mg/ml	27.633 ± 0.711	67.477 ± 0.826	39.996 ± 2.508	18.099 ± 2.970
1 mg/ml	95.228 ± 2.013	69.304 ± 0.832	78.140 ± 2.432	48.232 ± 3.851
2 mg/ml	84.897 ± 1.631	82.145 ± 0.055	34.339 ± 3.485	85.429 ± 2.970
4 mg/ml	66.320 ± 1.631	44.749 ± 1.065	22.583 ± 1.764	69.461 ± 1.485
Oxytocin (10 IU)	80.206 ± 2.497		65.672 ± 3.735	

*n* = triplicate observations, SEM: standard error of the mean.

**Table 2:** Summary of behavioural responses and general appearance of Wistar rats treated with single dose of *U. anisatum* root water extract in the acute oral toxicity study.

Observation	*Control group (physiological saline)*		*Experimental group*			
			*Single dose (300 mg/kg)*		*Single dose (2000 mg/kg)*	
	4 hrs	24 hrs	4 hrs	24 hrs	4 hrs	24 hrs
Skin colour change	Normal	Normal	Normal	Normal	Normal	Normal
Eye colour change	Normal	Normal	Normal	Normal	Normal	Normal
General physique	No effect	No effect	No effect	No effect	No effect	No effect
Diarrhoea	Unobserved	Unobserved	Unobserved	Unobserved	Unobserved	Unobserved
Coma	Unobserved	Unobserved	Unobserved	Unobserved	Unobserved	Unobserved
Drowsiness	Unobserved	Unobserved	Unobserved	Unobserved	Unobserved	Unobserved
Sedation	No effect	No effect	No effect	No effect	No effect	No effect
Gasping	Unobserved	Unobserved	Unobserved	Unobserved	Unobserved	Unobserved
Tremor	Unobserved	Unobserved	Unobserved	Unobserved	Unobserved	Unobserved
Salivation	Normal	Normal	Normal	Normal	Normal	Normal
Mortality	No death	No death	No death	No death	No death	No death

**Table 3:** Biochemical estimation of blood serum of Wistar rats at 14th day after treatment with the *U. anisatum* root water extract at the 2000 mg/kg dose level in the acute oral toxicity study.

Parameter	Normal range	Mean ± SEM of observed values at 0 mg/kg (control)	Mean ± SEM of observed values at 2000 mg/kg
ALP (IU/L)	20–256	134 ± 11.12	113.5 ± 1.5
ALT (IU/L)	28–132	199 ± 6.71	102.5 ± 3.5
AST (IU/L)	59–247	183.9 ± 17.7	179.0 ± 2.0
Urea (mmol/L)	3.2–7.5	6.92 ± 3.47	7.1 ± 0.9
Creatinine (*μ*mol/L)	4.0–57	23.13 ± 0.88	29.5 ± 0.5

*n* **=** duplicate observations, SEM: standard error of the mean.

**Table 4:** Toxic effect of the *U. anisatum* root water extract on some hematological parameters of Wistar rats on the 14th day.

Parameter	Normal range	Mean ± SEM of observed values on control rats (0 mg/kg)	Mean ± SEM of observed values on experimental rats (2000 mg/kg)
Neutrophils	10–40%	16.02 ± 3.42	17.0 ± 3.6%
Lymphocytes	55–95%	78. 32 ± 1.76	81.0 ± 4.7%
Eosinophils	0–4%	1.13 ± 0.91	2.0 ± 1.15%
Basophils	0–1%	0%	0%

*n* **=** duplicate observations, SEM: standard error of the mean.

**Table 5:** Phytochemical composition of *U. anisatum* root powder, water, and ethanol extracts.

Phytochemical class	Test	Powder	Ethanol extract	Water extract
Alkaloid	Mayer's	+	+	+
	Drangedorff's	+	+	+
Glycosides	Kedde	+	+	+
	Keller–Killiani	+	+	+
	Borntrager's	+	+	+
Saponins	Foam	+	+	+
Phytosterols	Lieberman	+	+	+
Triterpenes	Salkowski's test	+	+	+
Phenols	Ferric chloride	+	+	+
Flavonoids	Sodium hydroxide	+	+	+
Diterpenes	Copper acetate	+	+	+
Proteins	Xanthoproteic	+	+	+
Fixed oils	Filter paper	+	+	+
Essential oils	Hydro distillation	+	ND	ND

+ present; − absent; ND: not done.

## Data Availability

All data underlying the results are available as part of the article and no additional source data are required.
